The article "APPL1-Mediating Leptin Signaling Contributes to Proliferation and Migration of Cancer Cells" was retracted in 2023. Reasons: duplicated images; unreliable data; concerns about the data.

# APPL1-Mediating Leptin Signaling Contributes to Proliferation and Migration of Cancer Cells

**DOI:** 10.1371/journal.pone.0166172

**Published:** 2016-11-07

**Authors:** Youming Ding, Yingkang Cao, Bin Wang, Lei Wang, Yemin Zhang, Deling Zhang, Xiaoyan Chen, Mingxin Li, Changhua Wang

**Affiliations:** 1 Department of Hepatobiliary & Laparascopic Surgery, Wuhan University Renmin Hospital, Wuhan, 430060, China; 2 Department of Pathology & Pathophysiology, Wuhan University School of Basic Medical Sciences, Wuhan, 430071, China; Duke University School of Medicine, UNITED STATES

## Abstract

Leptin has been implicated in tumorigenesis and tumor progression, particularly in obese patients. As a multifunctional adaptor protein, APPL1 (containing pleckstrin homology domain, phosphotyrosine binding domain, and a leucine zipper motif 1) plays a critical role in regulating adiponectin and insulin signaling pathways. Currently, high APPL1 level has been suggested to be related to metastases and progression of some types of cancer. However, the intercourse between leptin signaling pathway and APPL1 remains poorly understood. Here, we show that the protein levels and phosphorylation statues of APPL1were highly expressed in tissues from human hepatocellular carcinoma and triple-positive breast cancer. Leptin stimulated APPL1 phosphorylation in a time-dependent manner in both human hepatocellular carcinoma HepG2 cell and breast cancer MCF-7 cell. Overexpression or suppression of APPL1 promoted or attenuated, respectively, leptin-induced phosphorylation of STAT3, ERK1/2, and Akt in the cancer cells, accompanied with enhanced or mitigated cell proliferation and migration. In addition, we identified that APPL1 directly bound to both leptin receptor and STAT3. This interaction was significantly enhanced by leptin stimulation. Our results suggested that APPL1 positively mediated leptin signaling and promoted leptin-induced proliferation and migration of cancer cells. This finding reveals a novel mechanism by which leptin promotes the motility and growth of cancer cells.

## Introduction

A growing body of carefully executed epidemiological studies has highlighted associations between obese subjects and increased risk of several cancer types including hepatocellular carcinoma (HCC) and breast cancer [1–5]. Leptin is produced by the fat tissue and is a biomarker of obesity[6]. Indeed, high leptin levels are found in both animal models of obesity and obese individuals. Through binding to its receptor, leptin stimulates a cascade of signaling events and elicit subsequent cellular effects such as regulating adiposity, energy balance, and endocrine function as well as immune reaction. In the past decades, leptin has also been shown to play an essential role in tumorigenesis, tumor progression, and metastasis, due to its oncogenic, mitogenic, pro-inflammatory, and pro-angiogenic actions [7–10]. Thus, the molecules in leptin signaling pathway have become ideal drug targets for the prevention and treatment of various types of cancer, especially in obese patients [7, 11].

The article "APPL1-Mediating Leptin Signaling Contributes to Proliferation and Migration of Cancer Cells" was retracted in 2023. Reasons: duplicated images; unreliable data; concerns about the data.

APPL1 (adaptor protein, phosphotyrosine interaction, PH domain and leucine zipper containing 1) is a multi-functional adaptor protein mediating adiponectin function and potentiating insulin signaling [12–14]. Currently, APPL1 protein was found to be highly expressed in some tumor tissues such as aggressive prostate cancer tissues [15, 16]. Silencing of APPL1 resulted in a decrease in TGFβ-induced invasion of both human prostate cancer PC-3U cells and breast carcinoma MDA-MB-231 cells [15]. In addition, APPL1 depletion significantly enhanced the radiosensitivity of pancreatic cancer cells [17]. These data strongly suggest that APPL1 plays a critical role in cancer growth under certain physiological and pathophysiological circumstances. However, the underlying mechanism remains poorly understood.

We here report that APPL1 was highly expressed in human hepatocellular carcinoma and triple-positive breast cancer. We also found that leptin stimulated APPL1 phosphorylation in both HepG2 and MCF-7 cancer cells. Importantly, APPL1 mediated leptin signaling through binding with leptin receptor and STAT3. Overexpression or suppression of APPL1 promoted or attenuated, respectively, leptin-induced proliferation and migration of cancer cells. Our results provide the first evidence that APLL1 levels are tightly linked to leptin-induced proliferation and migration of cancer cells.

## Materials and Methods

### Reagents

The primary antibodies used in this study were obtained from Cell Signaling Technology (Beverly, MA, UAS). Protein A-sepharose beads was purchased from Amersham-Pharmacia Biotech (Piscataway, NJ, USA). Human recombinant leptin (L4146) was procured from Sigma Chemical Co. (St. Louis, MO, USA). AG490 (658401), LY294002 (440206), PD98059 (513000), TWS119 (361554), and Gö 6976 (365250) were purchased from Calbiochem (San Diego, LA, USA).

### Clinical specimens

The independent diagnosis of each case was confirmed by both pathologists and physicians according to WHO criteria. The frozen tumor tissues and their paired adjacent non-tumor tissues were obtained from the Department of Clinic Pathology of Wuhan University Renmin Hospital. Written informed consent from the patients was obtained, and this series of studies was reviewed and approved by Institutional Ethics Committees of Wuhan University Renmin Hospital.

The article "APPL1-Mediating Leptin Signaling Contributes to Proliferation and Migration of Cancer Cells" was retracted in 2023. Reasons: duplicated images; unreliable data; concerns about the data.

### Cell cultures

Human hepatocellular carcinoma cell line HepG2 and human breast cancer cell line MCF-7 were purchased from American Type Culture Collection (ATCC, Rockville, MD, USA) and routinely cultured in Dulbecco’s Modified Eagle Medium (DMEM) supplemented with 10% FBS and 1% penicillin/streptomycin in the presence or absence of 0.1% amphotericin, respectively, in humidified atmosphere containing 5% CO_2_ and 95% air at 37°C.

### Virus infection

Serum-starved cells were infected with adenovirus carrying human full-length APPL1 or shRNA against human APPL1 (gifts from Drs. Feng Liu and Lily Q Dong, University of Texas Health Science Center at San Antonio, San Antonio, TX, USA) for 6 h and then cultured in complete medium for 36 h. Adenovirus carrying β-galactosidase or shRNA scramble sequences served as controls. After 42 h of infection, the cells were ready for experiments.

### Cell proliferation assay

Cell proliferation was confirmed by 3-(4,5-dimethylthiazol-2-yl)-2,5-diphenyltetrazolium bromide (MTT) assay and bromodeoxyuridine (BrdU) incorporation analysis, respectively. MTT assay was performed as our previously described protocol [18, 19]. BrdU assay was carried out using BrdU Cell Proliferation Assay Kit (#6813, CST, Danvers, MA, USA) according to the manufacturer’s instructions.

### Apoptosis determination

Apoptosis was induced by serum starvation for 60 h [20–22]. After treatment, the cells were fixed with 3.8% paraformaldehyde for 20 min, and then stained with the terminal deoxyribonucleotidyl transferase (TdT)-mediated dUTP-digoxigenin nick end labeling (TUNEL) reagent (Roche, Basel, Switzerland) for in situ apoptosis detection. Positive and negative controls were pretreated with 10 U/ml DNase or incubated without TdT, respectively. Apoptotic cells were detected under an Olympus FluoView FV1000 Confocal Microscope.

### Wound healing assay

Monolayer cells were grown to 100% confluence, created linear scratch wounds by using a pipette tip, and then treated with 100 nM leptin for 12 h. Mitomycin C (0.1 mg/ml) was added to inhibit cell proliferation. Photographs were taken immediately after wound induction and following 12 h incubation. The wound gap widths were measured using ImageJ software.

### Immunoprecipitation, western blot, and Pro-Q diamond phosphoprotein analysis

Total proteins were extracted by lysis buffer containing 50 mM HEPES (pH 7.5), 150 mM NaCl, 20 mM Na pyrophosphate, 10 mM NaF, 1 mM NaVO_3_, 2 mM EDTA, 10% glycerol, 1 mM MgCl_2_, 1 mM CaCl_2_, 10% Nonidet-P40, 2 mM PMSF, and 10% phosphorylase inhibitor cocktail-I, -II, and -III. Protein concentration was determined using BCA (bicinchoninic acid) Protein Assay Reagent (Thermo, Rockford, IL, USA). For immunoprecipitation, cell lysates were incubated overnight with specific antibodies bound to Protein A-sepharose beads at 4°C. After incubation, the beads were washed extensively with ice-cold wash buffer containing 50 mM HEPES, pH 7.6, 150 mM NaCl, and 0.1% Triton X-100. Proteins bound to the beads were eluted by heating at 95°C for 10 min in SDS-PAGE sample loading buffer. The proteins were separated by SDS-PAGE gel, transferred to a nitrocellulose membrane, and detected with specific antibodies. The quantification of the relative increase in protein expression and phosphorylation statuses was normalized with control protein expression in each experiment using Quantity One software (Bio-Rad, Philadelphia, PA, USA).

The article "APPL1-Mediating Leptin Signaling Contributes to Proliferation and Migration of Cancer Cells" was retracted in 2023. Reasons: duplicated images; unreliable data; concerns about the data.

Phosphorylation analysis for APPL1 was performed using Pro-Q Diamond phosphoprotein gel stain according to the manufacturer's protocol (Molecular Probes, Invitrogen, Carlsbad, CA, USA). In brief, APPL1 was immunoprecipitated and separated by SDS-PAGE gel. The levels of APPL1 were determined by western blot using specific anti-APPL1 antibody. Phosphoprotein bands were scan by fluorescence at 532 nm [23, 24].

### Statistical analysis

Data are presented as the mean ± SD. Differences were examined using one way ANOVA followed by Tukey–Kramer post-hoc test and independent samples *t*-test. Chi Square was used to test differences between two or more actual samples. P values less than 0.05 (*p*<0.05) were considered statistically significant. Each experiment *in vitro* was repeated at least 3 times with similar results.

## Results

### APPL1 protein and phosphorylation were highly expressed in human hepatocellular carcinoma and triple-positive breast cancer

Using western blot to analyze a series of paired human tumors and adjacent non-tumor tissues for the expression pattern of APPL1, we found that APPL1 was highly expressed in human hepatocellular carcinoma (HCC) and triple-positive breast cancer (TPBC) when compared with their matched non-tumor counterparts (Fig 1A and 1D), suggesting a positive correlation of APPL1 with tumorigenesis. By scoring 43 non-tumor tissues and 51 tumor tissues, we found that APPL1 abundances was significantly upregulated in 20.9% of non-tumor tissues and in 62.7% of HCC (*p*<0.01) (Fig 1B). Similar results were found in TPBC showing high expression of APPL1 in 19.5% of non-tumor tissues and in 80.4% of tumor tissues (Fig 1E). However, no relationship was observed between the APPL1 expression and other clinic pathological characteristics such as age, body weight, as well as stages (Data not shown). Given that APPL1 phosphorylation is associated with its function [12], we next investigated the phosphorylation statues of APPL1 in paired tumors and their adjacent non-tumor tissues and found that phosphorylated APPL1 highly existed in HCC and TPBC (Fig 1C and 1F). These results indicated that APPL1 protein levels and its phosphorylated statues were dramatically enhanced in tumor tissues.

The article "APPL1-Mediating Leptin Signaling Contributes to Proliferation and Migration of Cancer Cells" was retracted in 2023. Reasons: duplicated images; unreliable data; concerns about the data.

**Fig 1:** APPL1 levels in cancer tissues and phosphorylation in leptin-stimulated cancer cells. (**A**) Representative western blot images of APPL1 protein in paired hepatocellular carcinoma and their adjacent non-tumor tissues (n = 21). APPL1 levels were normalized to tubulin and quantitative analysis was represented in the bottom panel. (**B**) The percentage of APPL1 highly expressed cases in hepatocellular carcinoma and non-tumor tissues detected by western blot. (**C**) Representative western blot images of APPL1 phosphorylation in paired hepatocellular carcinoma and their adjacent non-tumor tissues (n = 21). Phosphorylated APPL1 were normalized to APPL1 protein and quantitative analysis was represented in the bottom panel. (**D**) Representative western blot images of APPL1 protein in paired triple-positive breast cancer and their adjacent non-tumor tissues (n = 21). APPL1 levels were normalized to tubulin and quantitative analysis was represented in the bottom panel. (**E**) The percentage of APPL1 highly expressed cases in triple-positive breast cancer and non-tumor tissues detected by western blot. (**F**) Representative western blot images of APPL1 phosphorylation in paired triple-positive breast cancer and their adjacent non-tumor tissues (n = 21). Phosphorylated APPL1 were normalized to APPL1 protein and quantitative analysis was represented in the bottom panel. (**G and H**) Representative western blot images and quantitative analysis of APPL1 phosphorylation in human hepatoma HepG2 cells (G) and breast cancer MCF-7 cells (H) under stimulation with leptin. Phosphorylated APPL1 were normalized to APPL1 protein and quantitative analysis was represented in the bottom panel. (**I**) Effects of PKC inhibitor Gö 6976 and GSK3β inhibitor TWS119 on leptin-stimulated APPL1 phosphorylation. *p<0.05, **p<0.01, ***p<0.001 *vs* the non-tumor group or control group. N: non-tumor tissue; T: tumor tissue.

### Leptin stimulated APPL1 phosphorylation

To study the impact of leptin on APPL1 phosphorylation, the cells were starved serum for 6 h and then treated with 100 nM leptin for 15, 30, or 60 min. We found that leptin administration significantly increased APPL1 phosphorylation in a time-dependent manner in human HepG2 hepatoma cells (Fig 1G) and MCF-7 breast cancer cells (Fig 1H). When serum-starved cells were pretreated with or without 10 μM PKC inhibitor Gö 6976 or 1 μM GSK3β inhibitor TWS119 for 1 h and then stimulated with or without 100 nM leptin for 30 min, we found that leptin-induced APPL1 phosphorylation remains unchanged in HepG2 cells and MCF-7 cells under concomitant treatment with Gö 6976 or TWS119 (Fig 1I). These results suggest that leptin-stimulated phosphorylation was independent on PKC and GSK3β.

The article "APPL1-Mediating Leptin Signaling Contributes to Proliferation and Migration of Cancer Cells" was retracted in 2023. Reasons: duplicated images; unreliable data; concerns about the data.

### APPL1 positively regulated leptin-induced proliferation and migration of cancer cells

To figure out the potential role of APPL1 in cancer growth, we tested its impacts on cell proliferation, apoptosis, and migration in HepG2 cells and MCF-7 cells. The cells overexpressing APPL1were cultured in serum-free DMEM for 6 h followed by exposure to 100 nM leptin for 24 h. MTT and BrdU assays were performed to valuate cell proliferation. As shown in Fig 2A and 2B, APPL1 overexpression significantly increased leptin-stimulated cell proliferation. When cancer cells were incubated in serum-free DMEM in the presence or absence of 100 nM leptin for 60 h, we found that APPL1 overexpression further enhanced anti-apoptosis ability of leptin (Fig 2C). We next used a wound-healing assay to determine the impact of APPL1 on cell migration. Monolayer cancer cells were grown to 100% confluence and then treated with 100 nM leptin for 12 h. Mitomycin C (0.1 mg/ml) was used to avoid potential effect of cell proliferation on migration. We found that overexpressed APPL1 markedly increased the wound healing abilitiy of leptin, as evidenced by a further increase in wound closure (Fig 2D). Using similar strategies, we found that APPL1 suppression by shRNA prevented leptin-induced changes in cell proliferation (Fig 3A and 3B), apoptosis (Fig 3C), and migration (Fig 3D). These results strongly suggest that APPL1 mediated the promotive effect of leptin on growth and migration of cancer cells.

**Fig 2:** Effect of APPL1 overexpression on leptin-stimulated proliferation and migration of cancer cells. (**A**) MTT assay in APPL1-overexpressing cancer cells. (**B**) BrdU incorporation assay in APPL1-overexpressing cancer cells. (**C**) Cell apoptosis determined by TUNEL assay in APPL1-overexpressing cancer cells. (**D**) Quantitative analysis of wound closure in APPL1-overexpressing cancer cells. (n = 4). *p<0.05, **p<0.01 *vs* indicated group.

**Fig 3:** Effect of APPL1 knockdown on leptin-stimulated proliferation and migration of cancer cells. (**A**) MTT assay in APPL1-silencing cancer cells. (**B**) BrdU incorporation assay in APPL1-silencing cancer cells. (**C**) Cell apoptosis determined by TUNEL assay in APPL1-silencing cancer cells. (**D**) Quantitative analysis of wound closure in APPL1-silencing cancer cells. (n = 4). *p<0.05, **p<0.01 *vs* indicated group.

The article "APPL1-Mediating Leptin Signaling Contributes to Proliferation and Migration of Cancer Cells" was retracted in 2023. Reasons: duplicated images; unreliable data; concerns about the data.

### APPL1 facilitated leptin signaling

To elucidate the molecular mechanism underlying APPL1 action, we examined whether altering APPL1 expression affects leptin-stimulated phosphorylation of STAT3, Akt, and ERK. The cells infected with adenovirus carrying full-length APPL1 or shRNA against human APPL1 were cultured in serum-free DMEM for 6 h and then stimulated with 100 nM leptin for 6 h. As expected, overexpression of APPL1 potentiated leptin-stimulated phosphorylation of STAT3, ERK1/2, and Akt in HepG2 cells and MCF-7 cell (Fig 4A–4D). In contrast, suppression of APPL1 impaired leptin-dependent phosphorylation of STAT3, ERK1/2, and Akt (Fig 5A–5D). These results confirm that APPL1 positively mediated leptin signaling.

**Fig 4:** Effect of APPL1 overexpression on leptin signaling in cancer cells. (**A**) Representative western blot bands of phosphorylation levels of signaling molecules in leptin signaling in APPL1-overexpressing cancer cells. (**B**) Quantitative analysis of phosphorylation levels of STAT3 in (A). (**C**) Quantitative analysis of phosphorylation levels of ERK1/2 in (A). (**D**) Quantitative analysis of phosphorylation levels of Akt in (A). (n = 3). *p<0.05, ** *p*<0.01 *vs* indicated group.

**Fig 5:** Effect of APPL1 konckdown on leptin signaling in cancer cells. (**A**) Representative western blot bands of phosphorylation levels of signaling molecules in leptin signaling in APPL1-silencing cancer cells. (**B**) Quantitative analysis of phosphorylation levels of STAT3 in (A). (**C**) Quantitative analysis of phosphorylation levels of ERK1/2 in (A). (**D**) Quantitative analysis of phosphorylation levels of Akt in (A). (n = 3). *p<0.05, **p<0.01 *vs* indicated group.

We next examined whether APPL1 interacts with signaling molecules of leptin signaling pathway. The cells were incubated with serum-free DMEM for 6 h and then treated with 100 nM leptin for 6 h. By *in vitro* pull-down studies, we found that APPL1 fused with glutathione S-transferase (GST) (GST-APPL1), but not GST alone, interacted with leptin receptor (LR) and STAT3 (Fig 6A). In addition, endogenous LR and STAT3 were coimmunoprecipitated with endogenous APPL1 in cancer cells (Fig 6B). This interaction was enhanced by leptin stimulation (Fig 6C and 6D). These data indicate that APPL1 physically interacted with both LR and STAT3.

**Fig 6:** APPL1 interacted with leptin receptor and STAT3 in cancer cells. (**A**) The glutathione S-transferase (GST) pull-down assay to detect the interaction between APPL1 and leptin receptor (LR) or STAT3. (**B**) Co-immunoprecipitation assay to detect the interaction between endogenous APPL1 and endogenous LR or STAT3. (**C and D**) Quantitative analysis of association between APPL1 and LR or STAT3 in HepG2 cells (C) and MCF-7 cells (D). (n = 3). **p<0.01, ***p<0.001 *vs* indicated group.

The article "APPL1-Mediating Leptin Signaling Contributes to Proliferation and Migration of Cancer Cells" was retracted in 2023. Reasons: duplicated images; unreliable data; concerns about the data.

### Concomitant activation of the JAK/STAT3, PI3K/Akt, and ERK signaling was responsible for proliferation and migration of cancer cells

To figure out signal transduction pathways plausibly involved in APPL1-mediating leptin action, the cells overexpressing APPL1 were serum-starved for 6 h and then pretreated with 100 μM AG490 (a specific and potent inhibitor of JAK2), 10 μM PD98059 (a potent and selective inhibitor of ERK1/2), or 10 μM LY294002 (a specific inhibitor of PI3K/Akt pathway) for 1 h followed by treatment with 100 nM leptin for another 6 h (for western blot) or 24 h (for MTT and BrdU assays). As shown in Fig 7, blocking these pathways significantly inhibited leptin-induced stimulation of proliferation (Fig 7B and 7C), when compared with leptin treatment alone. In addition, inhibition of these pathways also significantly increased cell apoptosis (Fig 7D) and reduced cell migration (Fig 7E). Interestingly, leptin-stimulated phosphorylation of both ERK1/2 and Akt was suppressed by AG490 treatment whereas leptin-stimulated STAT3 phosphorylation was not affected by treatment with PD98059 or LY294002 (Fig 7A), suggesting that STAT3 was an upstream kinase for both ERK1/2 and Akt.

**Fig 7:** Effect of inhibitors of JAK/STAT3, ERK, or Akt signaling pathway on leptin-stimulated proliferation and migration of APPL1-overexpressing cancer cells. (**A**) Representative western blot bands of phosphorylation levels of signaling molecules in leptin signaling. (**B**) MTT assay. (**C**) BrdU incorporation assay. (**D**) Cell apoptosis determined by TUNEL assay. (**E**) Quantitative analysis of wound closure. (n = 3). *p<0.05, **p<0.01 *vs* indicated group.

## Discussion

The previous studies have shown that APPL1 protein promotes invasion and progression of some cancer types by altering early endosome biogenesis [16, 25], provoking alternative TGFβ signaling pathways [15], modulating DNA repair [17], or promoting cell cycle progress [26]. In the present study, we found a novel mechanism of APPL1-directed proliferation and migration of cancer cells by positively regulating leptin signaling pathway.

We observed the increased APPL1 protein levels in human HCC and TPBC (Fig 1A and 1D), which is consistent with previous studies showing that APPL1 protein is high expressed in prostate cancer [15, 16]. Moreover, we found that APPL1 phosphorylation was significantly increased in cancer tissues when compared with adjacent non-tumor tissues (Fig 1C and 1F). Given that APPL1 phosphorylation is critical for its function [12], our results supported a possibility of that APPL1 may influence the growth of human HCC and TPBC. However, no significant difference was found among APPL1 levels, body mass index (BMI), metastases, and pathological grade (Data not shown), due to limited clinical specimens in this study. Future studies in larger clinical materials are needed to evaluate the clinical value of APPL1 as a potential cancer prognostic marker, particularly in patients with obesity or type 2 diabetes mellitus.

The article "APPL1-Mediating Leptin Signaling Contributes to Proliferation and Migration of Cancer Cells" was retracted in 2023. Reasons: duplicated images; unreliable data; concerns about the data.

Previous studies have evidenced that APPL1 undergoes phosphorylation at Ser(430) in the liver tissues and hepatocytes, and at Ser (401) in C2C12 cells, mediated by ER stress-induced PKCα or leptin-stimulated GSK-3β, respectively [27, 28]. In the present study, we found that leptin administration increased APPL1 phosphorylation in a time-dependent manner in the cancer cells (Fig 1G and 1H). Due to lack of commercial phosphor-APPL1 antibodies, phosphorylation analysis for APPL1 was performed using Pro-Q Diamond phosphoprotein gel stain in the present study [23, 24, 29, 30]. Our results just showed that the total phosphorylation statues of APPL1 but no phosphorylation of specific residues in APPL1 was enhanced by leptin stimulation. Interestingly, we found that pharmacological inhibition of either PKCα or GSK3β did not significantly affect total phosphorylation statues of APPL1 (Fig 1I), suggesting that leptin-stimulated APPL1 phosphorylation was independent on activities of PKCα and GSK3β in HepG2 cells and MCF-7 cells.

It has been well known that leptin is capable of promoting an aggressive cancer phenotype by stimulating growth, migration and invasion, and enhancement of angiogenesis in both normal and tumor cells including hepatocellular carcinoma and breast cancer [9, 31–34]. In agreement with this view, we found that leptin-induced proliferation and migration of cancer cells were promoted by overexpression of APPL1 (Fig 2), but attenuated by suppression of APPL1 (Fig 3), strongly suggesting that APLL1 positively regulated leptin-induced proliferation and migration of cancer cells.

Leptin activation of STAT3, AKT, and ERK1/2 signaling pathways has been suggested to be responsible for pro-cancer effect of leptin [7, 9]. In the present study, we found that overexpression of APPL1 significantly enhanced but APPL1 depletion abolished leptin-stimulated phosphorylation of STAT3, AKT, and ERK1/2 in cancer cells (Figs 4 and 5), suggesting that APPL1 mediated leptin signaling. In agreement with this view, inhibition of these pathways by specific inhibitors abrogated impact of APPL1 on stimulation of proliferation and migration of cancer cells by leptin (Fig 7). In addition, our findings showed that treatment of cancer cells with specific JAK/STAT3 inhibitor AG490 blocked leptin-stimulated phosphorylation of both ERK1/2 and AKT, whereas pharmacological inhibition of either ERK1/2 or Akt pathway did not affect leptin-induced STAT3 phosphorylation (Fig 7A), suggesting that activation of JAK/STAT3 was upstream of the activation of the ERK1/2 and AKT pathways [35].

The article "APPL1-Mediating Leptin Signaling Contributes to Proliferation and Migration of Cancer Cells" was retracted in 2023. Reasons: duplicated images; unreliable data; concerns about the data.

APPL1 is a multifunctional adaptor proteins located in the nucleus, endosome, and cytosol in various cells [36, 37]. Previous studies have shown that APPL1 associates with various signaling molecules [12, 23] and facilitate endocytosis of various receptors [38, 39]. We found that GST-fused APPL1 interacted with both leptin receptor and STAT3 (Fig 6A). In addition, we also confirmed that endogenous APPL1 co-immunoprecipitated with both endogenous leptin receptor and endogenous STAT3 in cancer cells (Fig 6B), and the interactions were dramatically enhanced by leptin stimulation (Fig 6C and 6D). These data suggest that APPL1 directly bound to leptin receptor and STAT3. Importantly, both leptin receptor and STAT3 localize at steady state in endosomes [40, 41]. Thus, it is plausible that APPL1 provide platforms for leptin-activated downstream signaling pathways or that the APPL1-associated endosomes play a role in regulating leptin signaling.

In conclusion, our study has identified APPL1 as a binding partner of leptin receptor and STAT3 protein. We have also evidenced that increased level of APPL1 could enhance leptin signaling pathways leading to cancer growth and progression. This finding reveals a novel mechanism by which leptin promotes the motility and invasiveness of cancer cells.
